# Neuronal Differentiation Dictates Estrogen-Dependent Survival and ERK1/2 Kinetic by Means of Caveolin-1

**DOI:** 10.1371/journal.pone.0109671

**Published:** 2014-10-28

**Authors:** Floriana Volpicelli, Massimiliano Caiazzo, Bruno Moncharmont, Umberto di Porzio, Luca Colucci-D’Amato

**Affiliations:** 1 Department of Pharmacy, University of Naples “Federico II”, Naples, Italy; 2 Institute of Genetics and Biophysics “Adriano Buzzati Traverso”, CNR, Naples, Italy; 3 Ecole Polytechnique Fédérale de Lausanne (EPFL), Lausanne, Switzerland; 4 Department of Medicine and Health Sciences, University of Molise, Campobasso, Italy; 5 Department of Environmental, Biological and Pharmaceutical Sciences and Technologies, Second University of Naples, Caserta, Italy; 6 C.I.R.N., Inter-University Center for Research in Neuroscience, Naples, Italy; II Università di Napoli, Italy

## Abstract

Estrogens promote a plethora of effects in the CNS that profoundly affect both its development and mature functions and are able to influence proliferation, differentiation, survival and neurotransmission. The biological effects of estrogens are cell-context specific and also depend on differentiation and/or proliferation status in a given cell type. Furthermore, estrogens activate ERK1/2 in a variety of cellular types. Here, we investigated whether ERK1/2 activation might be influenced by estrogens stimulation according to the differentiation status and the molecular mechanisms underling this phenomenon. ERK1/2 exert an opposing role on survival and death, as well as on proliferation and differentiation depending on different kinetics of phosphorylation. Hence we report that mesencephalic primary cultures and the immortalized cell line mes-c-myc A1 express estrogen receptor α and activate ERK1/2 upon E_2_ stimulation. Interestingly, following the arrest of proliferation and the onset of differentiation, we observe a change in the kinetic of ERKs phosphorylation induced by estrogens stimulation. Moreover, caveolin-1, a main constituent of caveolae, endogenously expressed and co-localized with ER-α on plasma membrane, is consistently up-regulated following differentiation and cell growth arrest. In addition, we demonstrate that siRNA-induced caveolin-1 down-regulation or disruption by means of ß-cyclodextrin treatment changes ERK1/2 phosphorylation in response to estrogens stimulation. Finally, caveolin-1 down-regulation abolishes estrogens-dependent survival of neurons. Thus, caveolin-1 appears to be an important player in mediating, at least, some of the non-genomic action of estrogens in neurons, in particular ERK1/2 kinetics of activation and survival.

## Introduction

In the central nervous system (CNS) a number of molecules contribute to the correct execution and maintenance of neural cells functions. Among these, the estrogens (E_2_), belonging to the family of steroid hormones, represent a critical class [1], [2].

It is well established that E_2_, as well as other steroids, mediates numerous actions in the CNS ranging learning to memory and neuroprotection [3], [4]. Moreover, they influence the fate of neural stem/progenitor cells when the cells are poorly supplied with mitogens or differentiation factors during the early stage of neurogenesis [5].

Indeed, E_2_ exert a dual role in proliferating and in non-proliferating cells. In proliferating cells, including glial cells in the CNS and in granule hippocampal neuron, E_2_ may foster cell proliferation and thus influence the neurogenesis in the dentate gyrus [6], [7], [8], [9]. On the other hands, E_2_ can exert a potent neuroprotective role influencing the survival of non-proliferating terminally differentiated neural cells *in* *vitro* [10]. In *vivo*, E_2_ also show neuroprotective antinflammatory role in different physiological and pathologic conditions including Parkinson’s and Alzheimer diseases, multiple sclerosis, and ischemic stroke [11], [12], [13], [14]. Two classical receptors, the estrogen receptor α and ß (ERα, ERß), are known to mediate the effects of E_2_. E_2_ binds the ER to activate or repress gene expression and this involves both genomic and non-genomic pathways. Genomic pathways include the classical interactions of ligand-bound ER dimers with estrogen-responsive elements in target gene promoters. The “genomic” effects are delayed in the onset and prolonged in duration. The “non-genomic” mechanism of E_2_ action has been only partially unraveled. It involves the activation of important signaling cascades including extracellular signal-regulated kinases 1/2 (ERK1/2) and elicits effects that are rapid in onset and short in duration. These effects can be mediated by receptors located in or close to the plasma membrane, which can be the same ERα or ß and/or a novel ER subtype [15], [16], [17]. It has been shown a link between the caveolae and ERα. In some cell types caveolae are the site where ERα triggers the non-genomic signalling [18]. Caveolae are small non-clathrin coated invaginations of plasma membrane in the lipidic raft, organized by the membrane spanning protein caveolin-1 (Cav1). The caveolae are often described as signaling regulators that orchestrates the interaction of receptors and signaling molecules, modulating transmembrane signaling in a rapid and specific manner [19]. Moreover, recent findings have also implicated Cav1 in neuronal plasticity [20], [21], while Cav1 KO mice show a neuropathological phenotype similar to accelerated aging and Alzheimer’s disease [22].

It is worth noting that non-genomic mechanisms have been shown to be responsible, at least partly, for the neuroprotective effects ascribed to E_2_ [23]. Moreover, the effects of E_2_ and their mechanisms of actions appear to be cell context-specific and vary from cell proliferation, to differentiation, migration or cell death, in although, the molecular events underlying these non-genomic effects and neuronal survival and protection are still poorly understood.

Here we address the issue of the different E_2_ responses depending on the status of cell differentiation, in particular we describe the activation of ERK1/2 signaling and the role of Cav1 in the molecular mechanism(s) of cell survival using an immortalized mesencephalic cell line A1 (Mes-c-myc A1**)** or midbrain primary cultures (mesPC). A1 cells and mesPC can be grown under proliferating/undifferentiated or non-proliferating/differentiated conditions. Neurite outgrowth, neuronal electrophysiological properties and an increase of neuronal markers upon differentiation are observed [24], [25], [26], [27], [28].

## Materials and Methods

### A1 cell line growth

As previously described, A1 cell line was generated from our group by c-myc retroviral infection of mesencephalic primary cultures generated from 11-day-old mouse embryos and selected by neomycin resistance [24], [26]. Briefly A1 cells were cultured in proliferating conditions in Minimum Essential Medium and F12 medium (MEM/F12, Invitrogen, Milan, Italy) supplemented with 10% FBS (HyClone, Milan, Italy) or differentiated in serum free medium and in the presence of 1 mM cAMP (Sigma, Milan, Italy) and N2 supplement (Invitrogen).

### COS-7 cell line

COS cell is a fibroblast-like cell line derived from the CV-1 cell line by transformation with an origin defective mutant of SV40 which codes for wild type T antigen commercially available by ATCC. COS-7 were cultured in DMEM (Invitrogen) supplemented with 10% FBS (HyClone).

### Ethics Statement

All procedures involving mice were carried out in strict accordance with national and European safety and ethical rules and regulations according to the Council Directive 2010/63/UE (published on September 22th 2010) regarding the protection of animals used for experimental and other scientific purposes, as well national legislations (i.e., Italian Legislative Decree N° 116/92 and Italian Legislative Decree N° 388/98). C57BL/6J mice obtained from the Charles River Laboratories Italia s.r.l. (Milan, Italy) were housed in the animal facility of the Institute of Genetics and Biophysics under a 12-h light-dark schedule at a constant temperature and with food and water ad libitum. According to ethical responsibilities and 3R principles, all efforts were made to minimize animal suffering and to reduce the number of animals used (three or four for each experiment). Embryonic age (E) was determined by considering the day of insemination (as confirmed by vaginal plug) as day E0. Animals were sacrificed humanely, by putting mice into a box containing an increasing dose of CO_2_. Primary mesencephalic cultures were prepared from 11 or 13-day-old embryos as described below. E11 or E13 embryos were quickly removed and placed in PBS without calcium and magnesium and supplemented with 33 mM glucose. The ventral midbrain was carefully dissected under a stereoscope in sterile conditions and processed for cell cultures.

### MesPC cultures

Mouse ventral midbrain dissected from E11 embryos was dissociated using mechanical trituration with a fire polished Pasteur pipette in culture medium (see below) containing 0.01% pancreatic deoxyribonuclease (Sigma, Milan, Italy). As described dissociated cells were centrifuged, suspended in plating medium, counted and plated at a density of 40.000/cm^2^ [27], [28]. Proliferating cells were grown for 6 days in *vitro* (DIV) in the absence of serum with the addition of B27 supplement (Invitrogen), bFGF, (20 ng/ml, Sigma), FGF-8, (10 ng/ml) and the N-terminal fragment of the SHH protein (50 ng/ml). Differentiated cells were grown for 6 DIV as previously described and for additional 6 DIV in the absence of mitogens. Half of the medium was changed every three days.

### Estrogen stimulation

For E_2_ (Sigma) stimulation, A1 cells or mesPC were serum starved for 24 hrs and then treated with 10 nM E_2_ (Sigma) alone or in combination with 10 µM of the estrogen antagonist ICI 182 780 (Zeneca Ltd., London, England) or 10 mM of Methyl-ß-cyclodextrin (Sigma). Cultures were stimulated with E_2_, ICI 182–780, or ethanol 20% for different times as indicated in the figures. At the end of the incubation time, cells were washed three times with ice-cold PBS pH 7.4 and lysed as described (see below). Experiments with A1 cells or mesPC were always carried at least in triplicate sister samples for each experimental point analyzed.

### Western blot analysis

Western Blot analysis was carried as previously described [27]. Following the appropriate treatments and washing three times with ice-cold PBS, the A1 cells and the mesPC were harvested in lysis buffer (50 mM Hepes, 150 mM NaCl, 1 mM EDTA, 1 mM EGTA, 10% glycerol, 1% Triton X-100, 1 mM PMSF, 2 mM sodium orthovanadate, 5 mM sodium pyruvate, 10 mM sodium fluoride, protease inhibitors cocktails). The lysates were incubated 30 min on ice, and then clarified by centrifugation at 8000 g×10 min. Total protein concentration was estimated by modified Bradford assay (Bio-Rad, Milan, Italy). 50 µg/lane of total proteins were separated on 10% SDS polyacrylamide gel and then proteins were transferred to polyvinylidene difluoride (PVDF) membranes (Immobilon-P, Millipore Corporation, Milan, Italy); complete transfer was assessed using pre-stained protein standards (Bio-Rad). The membranes were blocked in TBS 1x (10 mM Tris, pH 7.4, 150 mM NaCl) and 5% non-fat powdered milk for 2 hr at room temperature (RT). Incubation with the primary antibody was carried out at RT for 2 hr. Finally, the membranes were incubated with the horseradish peroxidase-conjugated secondary antibody (1∶2500) for 2 h at RT and the reactions detected with ECL system (Amersham, Milan, Italy).

### Antibodies

Antibodies were purchased from the following sources: polyclonal anti Phospho-p44/42 MAP kinase (Thr202/Tyr204) antibody (New England Biolabs, Milan, Italy 1∶500); polyclonal anti ERK1/2 antibody (New England Biolabs, 1∶1000), rabbit anti-ERα (1∶500, SantaCruz, Milan, Italy); polyclonal anti caveolin-1 antibody (BD laboratories, Milan, Italy 1∶500).

### Transfection of mouse anti-Cav1 silencing oligonucleotides

In preliminary experiments we found that low cell density was a critical point for efficient RNA interference. Therefore we could not use the mDA cultures treated with bFGF for these experiments, because of the high cell proliferation. Thus we used primary cultures generated from an E13 mouse midbrain plated in serum-free NBM supplemented with B27 at a density of 100 000/cm^2^. After 5 days *in* *vitro* (DIV) non-proliferating*/*differentiated mesPC and A1 cells were transfected using Lipofectamine 2000 (Invitrogen), according to the manufacturer’s instructions. Briefly 50 nM of ON-TARGET plus SMART pool (L-058415, Dharmacon, Inc, Lafayette, Co, USA) siRNA construct targeting Cav1 or scrambled non-targeting siRNA (negative control; cat # D-001210-01-05, Dharmacon) was diluted in appropriate amount of Opti-MEM I medium (Invitrogen) without serum and mixed gently. At the same time appropriate amount of Lipofectamine 2000 was diluted in same medium, mixed gently and incubate for 5 minutes at RT. After incubation, the two solutions were combined and incubated for 20 minutes at RT to allow complex formation to occur. The complex was added to the cells and incubated at 37°C in CO_2_ incubator for 4 hr. After 4 hr culture medium was replaced with 10 nM of estrogen or vehicle for 48 hr.

### Immunocytochemistry and confocal microscopy

Cell cultures were fixed for 30 min at RT, in 4% paraformaldehyde in PBS, followed by three washes in PBS, permeabilized for 15 min in PBS containing 0.1% Triton X-100 and 10% normal goat serum (NGS) and incubated for 2 hr at RT or overnight at 4°C in the primary antibodies diluted in PBS containing 10% NGS. The following antibodies were used at the indicated dilutions: monoclonal (mAb) anti-Cav1 (BD laboratories, 1∶200), rabbit anti-ERα (1∶500, SantaCruz). After rinsing in PBS, the cells were incubated in fluorescent-labeled secondary antibodies (Texas red goat anti-rabbit, 1∶200, Invitrogen; goat anti-mouse fluorescein-conjugated, 1∶200, Chemicon, Milan, Italy) in PBS containing 5% NGS. Control cells were incubated in the same solutions without primary antibodies and subsequently processed as above. Three culture wells were analyzed in each experiment for every experimental condition. Images were acquired with laser scanning confocal microscopy (Fluorescence Inverted Confocal Microscope equipped with acquisition and processing software LEICA SP2 AOBS) and serial sections of the same specimen (“Z stacks”) were made in order to provide three-dimensional images and co-localization information. In the Z0 images of confocal stacks, acquired from different fields of proliferating or differentiated A1 cells were processed. Polygons representative of the cell image were delimited and numerical data relative to their pixels were analyzed. We considered positive pixels those with an intensity value >100 for estrogen receptor in the green channel and for Cav1 in the red channel. The percentage was calculated as the number of double positive pixels/estrogen positive pixels×100.

### RNA isolation and Real time PCR

Total RNA was isolated from A1 and mesPC cells using Tri-Reagent (Sigma) according to the manufacturer’s instructions. The analyses were always carried out in triplicate samples for each experimental point analyzed and were processed separately. The yield and integrity of RNA were determined by spectrophotometric measurement of A_260_ and agarose gel electrophoresis respectively. Briefly, 2 µg of RNA were reverse transcribed, using random hexanucleotides (New England Biolabs 6 mM) and 200 U of Moloney-murine leukemia virus reverse transcriptase (New England Biolabs). Gene specific primer sets (*Bnip 2* – Fw ACCCCTCTTGGTTTATCCGAA - Rw CTCGGCCAAGTTAAAGACGTA; *Prothymosin α* – Fw CTGCCAATGGGAACGCTCA - Rw TCCTCCTCACCGTCACCT; *Caveolin-1* - Fw CGACCCCAAGCATCTCAACGA - Rw CCTTCCAGATGCCGTCGAA) used for quantitative real time PCR (qRT-PCR, Applied Biosystem, Milan, Italy) were designed using OLIGO 6 software according to manufacturer’s instructions, in order to obtain amplified fragments with comparable length (around 120 bp). SYBR Green qRT-PCR reactions were performed in 96-well plates using 7900 HT Fast *Real*-*Time* PCR System (Applied Biosystem). Thermal cycling conditions comprised initial steps at 50°C for 2 minutes and 95°C for 10 minutes, followed by 40 cycles at 95°C for 15 seconds and 60°C for 1 minute. All samples were run in triplicate. Amplification efficiency of each primer pair was verified by performing qRT-PCR using different template dilutions. Gene expression levels were quantified from real-time PCR data by the comparative threshold cycle (*CT*) method using hypoxanthine phosphoribosyl transferase (HPRT) as an internal control gene. The fractional number of PCR cycles *CT* required to obtain a given amount of qRT-PCR product in the exponential phase of amplification was determined for the gene of interest and for HPRT in each RNA sample. The relative expression level of the gene of interest was then expressed as 2^−Δ*CT*^ where Δ*CT* = *CT* gene of interest - *CT* HPRT [29].

### MTT assay

Cell viability was analyzed using the 3-(4,5-dimethylthiazol-2-yl)-2,5-diphenyltetrazolium bromide (MTT) reagent assay according with the manufacturer’s instructions (Sigma). Briefly, the cells with 0,5 mg/ml of MTT were incubated at 37°C in a humidified 5% CO_2_/95% air mixture for 4 h. At the end of the incubation the cells were lysed with an equal amount of MTT solubilization solution (10% Triton X-100 in 0.1 N HCl in acid isopropanol). The optical density of each sample was measured with spectrophotometer (Beckmann Coulter, Milan, Italy) at 570 nm and subtracted background at 690 nm. All of the experiments were performed in triplicate.

### Tripan blue assay

Trypan Blue is a method used to analyze cell vitality. It is based on the principle that viable cells do not take up the dye, whereas dead cells incorporate it. The cell density was determined using a hemacytometer. Each square of the hemocytometer, with coverslip in place, represents a total volume of 0.1 mm^3^ or 10^4^ cm^3^. Since 1 cm^3^ is equivalent to approximately 1 ml, the subsequent cell concentration was determined using the following calculations: number of total cells = the average count per square×dilution factor×10^4^×volume. Viable cells (%) = [1.00–(Number of blue cells ÷ Number of total cells)]×100.

### Statistical analysis

For all experiments the analysis of variance was carried out, followed by post hoc comparison (ANOVA, Scheffè F-test). p<0.01 was considered statistically significant. Data were expressed as mean +/− SEM.

## Results

### A1 neural cells and mesPC as cellular models

To investigate the role of the Cav1 protein we used two cellular models: A1 cells and mesPC obtained both from mouse embryonic mesencephalon at day 11. The A1 cells, immortalized by the c-myc proto-oncogene, showed the presence of markers belonging to neural cell lineages [24], [25], [26]. By FACS analysis after serum starvation for 24 hrs, undifferentiated A1 cells were still proliferating and did not exit cell cycle (data not shown). Under these culture conditions the morphology appears flat and large and no neuritic processes could be observed. Upon serum withdrawal and cAMP stimulation, cells differentiate, arresting the cell cycle and undergoing morphological and neuronal differentiation with ensuing long neuritic processes and a birefringent cell body. In addition, they also display electrical properties, typical of neurons such as mature voltage-gated K^+^ and Na^+^ channels and show various neuronal markers [24], [25], [26]. Alternatively, we used the mesPC, grown in the absence of serum with or without addition of mitogens or morphogens such as basic fibroblast growth factor (bFGF), sonic hedgehog (SHH) and fibroblast growth factor 8 (FGF-8). As previously described by us and other groups, neuroblasts derived from ventral midbrain proliferate in the presence of bFGF. Under this culture conditions, virtually no glial cells are detectable and the neuroblasts actively proliferate. Upon bFGF, SHH and FGF8 withdrawal after 6 days *in* *vitro* (DIV) cell growth is arrested. These cultures express early neural marker and subsequently they show neurite outgrowth, expression of pan-neuronal markers such as light and medium neurofilament (NF-L, NF-M) and specific dopaminergic, GABAergic and glutamatergic neuronal markers [27], [28], [30].

### Caveolin-1 is highly expressed in A1 cells and in mesPC and increases upon differentiation and partly co-localizes with ERα on cell plasma membrane

To study whether the cell differentiation affected Cav1 and ERα expression, we performed western blot analysis on proliferating/undifferentiated and non-proliferating/differentiated A1 cells and mesPC (Figure 1). The ERα protein level in both cellular models did not change following the differentiation (Figure 1A, B). Protein extracts from COS cells transfected or untransfected with the full-length cDNAs of ERα, were used as positive or negative controls of the western blot, respectively (Figure S1A).

**Figure 1:** In A1 cells and in mesPC, differentiation increases Cav1 protein expression but not ERα. Lysates from A1 and from mesPC proliferating/undifferentiated and non-proliferating/differentiated were immunoblotted using ERα (A), Cav1 (B) and ß-actin (A, C) antibodies. ERα, Cav1 and ß-actin specific bands were detected at 67 kDa, 21 kDa and 42 kDa in both proliferating (prol.) and non-proliferating (diff.) cells. (B, D) The diagrams show the relative quantitation of the ERα and Cav1 in proliferating and non-proliferating A1 and in mesPC cell line respectively. Data are expressed as ratios of ERα/ß-actin and Cav1/ß–actin. The blots are representative of three separate experiments. Asterisks represent p<0.01 when compared to proliferating cultures (ANOVA, Scheffè F-test).

Furthermore to investigate whether the Cav1 protein level could be affected during the differentiation, we performed western blot analysis on proliferating and non-proliferating A1 cells and mesPC (Figure 1C, D). Cav1, as previously described, besides being an essential structural organizer of the caveolae, play an important role in the signal transduction and it has been shown to affect ERs signaling. Cav1 was expressed in A1 cells and its levels show a three-fold-increase upon differentiation. Similarly to A1 cells, mesPC neuroblasts also show a two-fold-increase of Cav1 protein when their proliferation is arrested and differentiation is triggered (Figure 1C, D).

As positive and negative controls we used COS cells transfected with a c-DNA encoding Cav1 or untransfected cells, respectively (Figure S1B).

We considered that a reciprocal distribution of ERα and Cav1 could take place on cell membrane and in order to investigate whether it changed before and after differentiation we used immunofluorescence and confocal microscopy. As shown in Figure 2A, both Cav1 and ERα are localized on cell membrane of A1 cells, where they also partly co-localize as highlighted by the merge of the two signals (Figure 2A). Analysis of Z0 images of confocal stacks, acquired from different fields of proliferating and differentiated A1 cells, showed a higher percentage of co-localization of ERα and Cav1 in plasma membranes of the differentiated cells compared to proliferating cells (Figure 2B). Analysis of different Z–stacks showed that ERα is also localized within the cell (Figure S2). In the same way, Cav1 was also present in differentiated mesPC as assessed by the double staining with the neuronal marker, ß-III Tubulin (TuJ1), and partly co-localize on cell membrane with ERα (Figure S3).

**Figure 2:** Co-localization of Cav1 and ERα on A1 cell membrane increases upon differentiation. (A) Immunofluorescent detection shows a partial co-localization of ERα and Cav1 in A1 cells proliferating/undifferentiated (A1 prol.) and non-proliferating/differentiated (A1 diff.). (B) The analysis of Z0 images of confocal stacks, acquired from different fields of proliferating and non-proliferating A1 cells, shows a higher percentage of co-localization of ERα and Cav1 in plasma membranes of the differentiated cells compared to proliferating/non-differentiated cells. Scale bar equal 40 µm.

### Estrogens induce ERK1/2 phosphorylation with a kinetic that varies according to the proliferative/differentiation status both in A1 cells and in mesPC

The MAP kinase cascade is implicated in E_2_ action in a variety of cell types, including neuroepithelial cells [31]. To analyze the effect of E_2_ on ERK1/2 phosphorylation we have stimulated proliferating and non-proliferating A1 cells with 10 nM of E_2_ for different times. By western blot analysis, in proliferating A1 cells we observed a 2.5-fold increase of ERK1/2 phosphorylation after 5 min of E_2_ treatment. Moreover, this phosphorylation reached a peak 15 min after E_2_ treatment and then decreased at the basal level after 60 min, remaining unchanged up to 120 min (Figure 3A, B). Interestingly, non-proliferating A1 cells showed a different kinetic of ERK1/2 phosphorylation, upon E_2_ stimulation. At 30 min, ERK1/2 phosphorylation showed 1.5-fold increase reaching a peak at 60 min and decreased to basal level after 120 min (Figure 3C, D). The specificity of E_2_ stimulation was demonstrated using E_2_ selective inhibitor (ICI 182–780). Undeniably its addition was able to prevent E_2_- dependent ERK1/2 phosphorylation (Figure 3).

**Figure 3:** In A1 cells, E_2_ induce ERK1/2 phosphorylation according to the proliferative/differentiation status. Western blot detection of p-ERK1/2 and ERK1/2 proteins in proliferating/undifferentiated (A) and non-prolifearting/differentiated A1 cells (C) treated at indicated time with 10 nM of E_2_ and 10 mM of ICI 182–780. Two specific bands were observed respectively at 44 and 42 kDa. Each blot is representative of three separate experiments. The diagrams show the relative quantitation of p-ERK1/2 and ERK1/2 in proliferating (B) and non-proliferating (D) A1 cells. Data are expressed as ratios of p-ERK1-2/ERK1-2. In diagrams are also showed the different trend lines of the kinetic of p-ERK following E_2_ stimulation. Asterisks represent p<0.01 when compared to control cultures treated with vehicle (ANOVA, Scheffè F-test).

To confirm whether E_2_ induces ERK1/2 phosphorylation with different kinetics that varies according to the proliferative/differentiation status we performed similar experiment in mesPC.

We showed that E_2_ stimulation in proliferating neuroblasts induced a progressive increase of ERK1/2 phosphorylation starting at 10 min, reaching the highest level after 240 min stimulation (Figure 4A, B). Differently, under non-proliferating conditions, we observed a sustained activation of p-ERK1/2 from 10 min up to 120 min and decreased after 240 min stimulation (Figure 4C, D).

**Figure 4:** In mesPC, E_2_ induces ERK1/2 phosphorylation according to the proliferative/differentiation status. Western blot detection of p-ERK1/2 and ERK1/2 proteins in proliferating (A) and non-proliferating mesPC (C) treated at indicated time with 10 nM of E_2_ and 10 mM of ICI 182–780. Two specific bands were observed respectively at 44 and 42 kDa. Each blot is representative of three separate experiments. The diagrams show the relative quantization of p-ERK1/2 and ERK1/2 in proliferating (B) and non-proliferating primary cells (D). Data are expressed as ratios of p-ERK1-2/ERK1-2. In diagrams are also showed the different trend lines of the kinetic of p-ERK1/2 following E_2_ stimulation. Asterisks represent p<0.01 when compared to control cultures treated with vehicle (ANOVA, Scheffè F-test).

Finally we also verify whether in A1 cells the E_2_-dependent genomic pathway can be activated using Real time PCR analysis of two genes whose expression is known to be dependent on genomic pathway, Bnip 2 and prothymosin α. We found that also genomic effects does occur in A1 cells upon E_2_ stimulation (Figure S4).

### ß-Cyclodextrin is able to change the kinetic of ERK1/2 phosphorylation following E_2_ administration in A1 cells

It has been shown that the caveolae and Cav1 are involved in E_2_ non-genomic signaling. In previous experiments we have found that the cell growth arrest and the differentiation were paralleled by an increase of Cav1 protein and a change of p-ERK1/2 kinetic both in A1 cells and in mesPC. Therefore, we used β-cyclodextrin, a drug known to interfere with the organization and the formation of caveolae, to assess whether p-ERK1/2 kinetic is affected by a redistribution of Cav1 on cellular membrane [32]. ß-cyclodextrin 10 mM for 60 min was able to cause a redistribution of Cav1 throughout the plasma cellular membrane of A1 cells (Figure S5). Subsequently, we have analyzed the kinetic of p-ERK1/2 upon E_2_ stimulation in A1 cells either untreated or treated with ß-cyclodextrin. As shown in Figure 5 the administration of β-cyclodextrin was able to change the kinetic of p-ERK1/2 in both proliferating (Figure 5A, B) and non-proliferating (Figure 5C, D) A1 cells. In particular, in proliferating A1 cells we observed ERK1/2 phosphorylation after 15 min of E_2_ stimulation when compared to the control, with a peak at 120 min (Figure 5A, B). In differentiated A1 cells, ERK1/2 phosphorylation increases after 30 min with a peak at 120 min (Figure 5C, D). Thus, ERK1/2 kinetic of phosphorylation showed a similar profile in proliferating and differentiating cells following ß-cyclodextrin administration.

**Figure 5:** In A1 cells the different kinetics of p-ERK1/2 activation are abolished by β-cyclodextrin administration. Western blot detection of p-ERK1/2 and ERK1/2 proteins in proliferating (A) and non-proliferating A1 cells (C) treated at indicated time with E_2_ and ß-cyclodextrin. Two specific bands were observed respectively at 44 and 42 kDa. Each blot is representative of three separate experiments. The diagrams show the relative quantization of p-ERK1/2 and ERK1/2 in proliferating (B) and non-proliferating (D) A1 cells. Data are expressed as ratios of p-ERK1-2/ERK1-2. The trend line shows the kinetic of p-ERK1/2 following E_2_ stimulation. Asterisks represent p<0.01 when compared to control cultures treated with vehicle (ANOVA, Scheffè F-test).

### Caveolin-1 silencing affects the ERK1/2-kinetic in mesPC and in A1 cells

To examine whether p-ERK1/2 kinetic induced by E_2_ stimulation was dependent on Cav1, we transfected differentiated mesPC and A1 with a pool of Cav1 specific siRNAs (siCav1). As control we used non-targeting sequences (NT). Real-time PCR and western blot analysis performed in mesPC cells showed 70% of Cav1 mRNA and a slightly lower Cav1 protein down-regulation compared to control cultures (Figure S6A, B). Similar results are obtained in A1 cells (Figure S6C, D).

In order to study whether p-ERK1/2 kinetic was affected by NT or siCav1 transfection we carried out western blot analysis in differentiated A1 and mesPC cells. In A1 cells, in the presence of NT sequence, upon E_2_ stimulation, p-ERK1/2 kinetic increased from 30 min up to 60 min with a peak at 60 min and decreased at 120 min (Figure 6A). This profile was similar to that described in Figure 3B.

**Figure 6:** Cav1 downregulation changes the kinetic of p-ERK1/2 activation in non-proliferating mesPC and A1 cells. Western blot detection of p-ERK1/2 and ERK1/2 proteins in non-proliferating A1 cells and mesPC transfected with ON-TARGET plus SMART pool, as a negative control (A, C) and Cav1 specific siRNAs (B, D) treated at indicated time with 10 nM of E_2_. Two specific bands were observed respectively at 44 and 42 kDa. Each blot is representative of three separate experiments. Data are expressed as ratios of p-ERK1-2/ERK1-2. Asterisks represent p<0.01 when compared to control cultures treated with vehicle (ANOVA, Scheffè F-test).

On the contrary, upon E_2_ stimulation, siCav1 transfection affected p-ERK1/2 kinetic, so that ERK1/2 phosphorylation increased after 15 min of E_2_ stimulation with a peak at 60 min and decreased at 120 min (Figure 6B).

Similarly, we performed the same experiment in mesPC. As shown in Figure 6C, upon E_2_ treatment, NT sequence did not affect p-ERK1/2 kinetic as previously described in Figure 4B: ERK1/2 phosphorylation, significantly increased from 10 min up to 120 min with a peak at 30 min and decreased at 240 min (Figure 6C). On the contrary, in the presence of Cav1 specific siRNAs, E_2_ stimulation induced an increase of ERK1/2 phosphorylation starting at 10 min and decreasing progressively between 60 min and 240 min (Figure 6D). Thus, Cav1 down-regulation affected the kinetic of ERK1/2 phosphorylation by anticipating the activation, shifting the peak and the amount of ERK1/2 phosphorylation.

### Caveolin-1 silencing affects E_2_ survival in mesPC and in A1 cells

To verify whether E_2_ stimulation had a pro-survival effect, A1 and mesPC cells were grown for 5 DIV in differentiation conditions. At 5 DIV, before E_2_ stimulation, MTT assay was performed (Figure 7) and in the same day, both A1 and mesPC cells were treated or not with E_2_ for successive 48 hr. So that control cultures at 5 DIV were compared with those at 7 DIV. As presented in Figure 7, MTT assay at 7 DIV shows a 25% decline in the cell survival. This effect was reduced by E_2_ treatment.

**Figure 7:** E_2_–dependent survival is affected by Cav1 downregulation. The diagrams show the E_2_ effect, assessed by MTT assay, in non-proliferating A1 (A) and mesPC (B) cells after transfection of non-targeting, NT, or Cav1 siRNA construct (siCav). P0 indicates the start point of E_2_ stimulation (5DIV). Asterisks represent p<0.01 when compared to control cultures treated with vehicle (ANOVA, Scheffè F-test). The hash sign represents p<0.05 between control cultures at 7DIV compared to control cultures at 5DIV (ANOVA, Scheffè F-test).

In order to evaluate whether the pro-survival effect of E_2_ occurs via Cav1, differentiated A1 and mesPC cells at 5 DIV were transfected with siCav1 or control sequence (NT). 4 hr upon transfection the cells were stimulated with 10 nM of E_2_ for 48 hr. At first, in order to rule out a toxic effect of NT and siCav1 siRNAs transfected cells were counted with trypan blue and compared to untransfected cell. No significant differences were observed (Figure S7).

Furthermore, we demonstrate that the pro-survival effect of E_2_ occurs via Cav1, by MTT experiment performed in A1 and mesPC cells. As shown in Figure 7, E_2_ stimulation significantly increases the survival of A1 and mesPC cells transfected with NT sequence. Our data indicate that E_2_ protection in both cell cultures was abolished in the presence of Cav1 siRNA. Therefore Cav1 down-regulation affects E_2_-mediated survival and strongly suggests that E_2_ survival is Cav1-mediated.

## Discussion

We used two mouse cellular models, namely the A1 cell line and mesencephalic primary cultures to characterize in neurons the presence of ERα and Cav1 in order to study some of the non-genomic effects exerted by E_2_ and the underlying mechanism(s). Either models, under appropriate culture conditions, exit cell cycle and undergo neuronal differentiation, thus allowing to address the issue of whether a different status of proliferation/differentiation can affect the non-genomic responses to E_2_. It is worth noting that in the chosen cellular models no bias due to the genetic background would interfere.

We have previously shown that A1 cells undergo differentiation upon serum withdrawal and cAMP stimulation and represent a veritable neural cell line [24]. In the present study we find that A1 cells express ERα either under undifferentiated/proliferating or differentiated/non-proliferating conditions. It is known that ERα is localized within the cells and acts as a dimer that binds to DNA at specific target sequences, the estrogen response elements, present in the promoter region of target genes. ERα is expressed in many cell types of different lineages. In the CNS, including the mesencephalon, ERα is present both on undifferentiated and differentiated neural cells where it is likely to exert different functions, by stimulating overlapping but also different substrates [33], [34]. The finding that in our cell line and primary culture models, ERα is expressed on both undifferentiated and differentiated cells, allows to study the biochemical mechanisms underlying the different effects exerted by E_2_ in the CNS according to differentiation.

It is well known that E_2_ can foster differentiation and proliferation of neural cells and also exert neuroprotection against noxious stimuli on different types of neurons either *in* *vitro* and *in* *vivo*. Since the discovery that in humans different ERs exist, inconclusive and sometimes conflicting data have been generated on the mechanism(s) underlying ERs biological effects, including differences exerted in undifferentiated and differentiated neural cells [17], [35], [36], [37]. It is likely that the inconclusiveness of the findings is due to the differences in experimental settings such as different cell types and different manner to trigger cell death and therefore different mechanisms of neuroprotection. Nevertheless, it as been undoubtedly proven that E_2_ protect brain damage via ERα and the protective mechanism(s) is independent on blood flow and it is likely to be due to effects exerted directly on neural cell [35].

Among different ERs, it is ERα to be prevalently found physically associated with Cav1 [38]. Moreover it has been described that E_2_-ERα complex preferentially activate ERK1/2 and PI3K/AKT pathway [38]. The non-genomic actions of E_2_ may play a role of particular importance in the CNS. For instance, E_2_ exert neurotrophic and neuroprotective actions and enhance synaptic plasticity [39]. Other important non-genomic effects involve proliferation and differentiation [31], [40].

Here, we have investigated an open issue regarding the molecular mechanism(s) by which non-genomic signaling cascades are activated by E_2_ and in particular in our cellular models we have demonstrated the link between the status of proliferation and differentiation and the different activation of ERK1/2. Caveolae are ω-shaped lipidic rafts [41], located on the plasma membrane of many cell types and organized by the membrane-spanning protein caveolins. In particular, Cav1 is a “multitasking” protein that participates in lipid and protein trafficking and regulates signal transduction. Although recent findings have shown a role of Cav1 in glutamate receptor signaling and LTP production little is known concerning the function/s of Cav1 in neurons. Its dysregulation in a number of diseases, such as neuronal injury, ischemia and Alzheimer’s disease suggests its involvement in pathological conditions [42], [43]. In particular, a recent analysis of Cav1 KO mice shows accelerated aging of neuronal cells with increased vulnerability to ischemic stress and loss of neuroprotection by ischemic preconditioning [22]. In addition, Cav1 deficient mice impair cell proliferation and decrease survival upon glucose restriction, causing impairment of mitochondrial function. Without Cav1, free cholesterol accumulates in mitochondrial membranes, increasing membrane condensation and reducing efficiency of the respiratory chain and intrinsic anti-oxidant defense. This mitochondrial dysfunction predisposes Cav1 deficient animals to mitochondrial related diseases such as neurodegenerative disease [44].

It is known that exogenous expression of Cav1 in cells lacking caveolae, results in the formation of mature invaginated caveolae while cells expressing the endogenous form of Cav1 always show the presence of caveolae [45], [46]. Thus it is likely that caveolar lipidic rafts are present on cell membrane of A1 cells since they express high levels of Cav1, part of which is localized on plasma membrane. Different laboratories have shown that caveolae and Cav1 are involved in E_2_ non-genomic signaling. In particular, Cav1 is involved in E_2_-dependent activation of ERK1/2 signaling in non-neuronal cells. Recently, data from Patel’s laboratory pointed towards a role of Cav1 in mediating ERK1/2 activation in primary neurons [22], [47], [48]. Our findings, taken together, show that in both cellular models, Cav1 and/or caveolae play a role in determining the kinetic of ERK1/2 activation upon E_2_ stimulation. In particular we demonstrate that i) ERα, at least in part, co-localizes on plasma cell membrane with Cav1 as seen by confocal microscopy; ii) differentiated/non proliferating cells present a consistent increase of Cav1 protein and display a different kinetic of ERKs stimulation as compared to undifferentiated/proliferating counterpart; iii) disruption of lipidic rafts/caveolae, by means β-cyclodextrin or siCav1, is able to change the kinetic of ERK1/2 phosphorylation upon to E_2_ stimulation; iv) Cav1 down-regulation changes the kinetic of ERK1/2 phosphorylation upon E_2_ stimulation; v) E_2_ stimulation needs Cav1 to mediate survival. Both ß-cyclodextrin or siCav1 experimental approaches have been used to perturb caveolae [49], [44]. In our experiments both of them are able to change the kinetic of ERKs phosphorylation although with a different profile. This is likely due to differences in the mechanisms of action of the two compounds, namely siRNA down-regulates protein expression whereas ß-cyclodextrin re-distributes the molecules within the cell.

Increasing evidence point towards a crucial role exerted by the kinetics of ERK1/2, more than its simple activation, in determining its biological effects. For instance, both in PC12 cells and in hippocampal neurons, ERK1/2 activation may alternatively lead to increased proliferation or to neuronal differentiation or to cell death depending on its kinetic of activation [50], [51], [52], [53]. It is tempting to speculate that the different kinetic of ERK1/2 activation observed in undifferentiated *versus* differentiated mesencephalic neural cells may, at least in part, account for the different effects that E_2_ play in developing and mature CNS or within adult brain among neurons at different stage of differentiation. The fact that in primary culture of embryonic mesencephalic neurons a different kinetic of ERK1/2 activation is also observed according to the proliferation condition further suggest that the processes of cell proliferation and differentiation may be important in dictating the kinetic of ERK1/2 activation in response to E_2_ by up-regulating Cav1 protein and increasing its membrane localization.

Recent findings show that ERK 1 and ERK2 might exert different actions, thus the ratio between the two isoforms may be of relevance [54]. Although in this paper we do not address such an issue, in our experiments, overall, either forms of ERK get phosphorylated upon E_2_ stimulation. It would be interesting to investigate the selective role of ERK isoforms by means of gain or loss of function experiments.

In our experimental settings E_2_ protect cells from death. It is well known that E_2_ exert a neuroprotective role also *in vivo* and in other *in* *vitro* cellular models. Our data also show that E_2_ needs Cav1 to mediate survival. To the best of our knowledge this is the first time that a link between E_2_, caveolin and cell survival has been shown in neuronal cells.

It is conceivable that in our *in* *vitro* models the process of differentiation and arrest of proliferation, by changing the expression and the localization of Cav1, modifies the mechanisms of cell survival and death and the kinetic of ERK1/2 activation. Actually we found that also genomic effects do occur in A1 cells upon E_2_ stimulation, as shown by Bnip 2 and prothymosin α expression [55]. Previous reports indicate that Cav1 may act both as a facilitator and a suppressor of cell death in different cellular context. For instance, in fibroblasts and epithelial cells Cav1 plays a proapoptotic role [56]. In multiple myeloma cells, cholesterol depletion by ß-cyclodextrin abrogates both IL-6 and IGF-1-dependent survival via negative regulation of Cav1 [57]. It remains to be established how the process of differentiation affects the formation, composition or the signaling properties of caveolae on neural cells. Future experiments will also clarify whether caveolae are involved also in the activation and/or in the kinetic of other signaling pathway stimulated by E_2_.

In conclusion, taken together our findings clarify the molecular mechanisms underlying the action of E_2_ on undifferentiated and differentiated neural cells without bias due to the genetic background and point towards Cav1 as an important player in mediating at least some of the non-genomic action of E_2_.

## Supporting Information

Figure S1 **Immunoblot blot analyses of ERΑ and Cav1 in A1 cells.** (A) The immunoblot blot detection of ERΑ shows a specific band of 67 kDa in both proliferating and differentiated A1 cells (lane 1 and 2) by comparison with controls (lane 3, positive control, protein extracts of COS cells transfected with ERΑ cDNA); lane 4, negative control, protein extracts from COS cells. (B) Western Blot analyzes of Cav1 shows a specific band of 21 kDa in both undifferentiated and differentiated A1 cells (lane 1 and 2) by comparison with controls (lane 3, positive control, protein extracts of FRT cells transfected with Cav1 cDNA, or not transfected with Cav1 cDNA, lane 4, negative control).
(TIF)

Figure S2 **ERα immunofluorescent detection in differentiated A1 cells.** Different Z-stacks show that ERα is localized both on cell membrane and within the cells. Scale bar equal 40 µm.
(TIF)

Figure S3 **Cav1, ERα and beta-III-tubulin immunofluorescent detection in differentiated mesPC cells.** Cav1 protein partly co-localizes on cell membrane with ERα in differentiated mesPC as assessed by merge.
(TIF)

Figure S4 **E_2_ induce genomic changes in A1 cells.** The diagrams show the mRNA levels of Bnip 2 and prothymosin α (protα) expression after treatment with 10 nM of E_2_, at time indicated in figure. Data are expressed as ratios of Bnip 2/Hprt and protα/Hprt. Asterisks represent p<0.01 when compared to control cultures treated with vehicle (ANOVA, Scheffè F-test).
(TIF)

Figure S5 **ß-cyclodextrin redistributes the amount of Cav1 on cellular plasma membrane.** Immunofluorescent detection of Cav1 in A1 cells untreated (A) and treated with 10 mM of ß-cyclodextrin for 1 h (B). Scale bar equal 80 µm.
(TIF)

Figure S6 **Evaluation of Cav1 down-regulation by Real Time PCR and western blot analysis in mesPC and A1 cells.** The diagrams show the Cav1 mRNA levels in mesPC (A) and A1 cells (C) transfected with a negative control (non-targeting, NT) or Cav1 siRNAs construct (siCav1). Data are expressed as ratios of Cav1/Hprt. Western blot analysis of Cav1 and ß-actin in mesPC (B) and A1 (D) cells transfected with NT or Cav1 siRNAs construct (siCav1). Cav1 and ß -actin specific bands were detected at 21 and 42 kDa respectively. Asterisks represent p<0.01 when compared to NT control (ANOVA, Scheffè F-test).
(TIF)

Figure S7 **Silencing transfection did not affect cell vitality.** A1 and mesPC differentiated cells, transfected with NT or siCav1 sequence or untransfected (control) were counted with trypan blue solution to assess cell viability. No significant differences were observed between transfected and untransfected cells.
(TIF)

## References

[1] McEwenBS (2010) Stress, sex, and neural adaptation to a changing environment: mechanisms of neuronal remodeling. Ann N Y Acad Sci 1204: E38–59.2084016710.1111/j.1749-6632.2010.05568.xPMC2946089

[2] MaggiA, CianaP, BelcreditoS, VegetoE (2004) Estrogens in the nervous system: mechanisms and nonreproductive functions. Annu Rev Physiol 66: 291–313.1497740510.1146/annurev.physiol.66.032802.154945

[3] TakayasuY, TakeuchiK, KumariR, BennettMV, ZukinRS, et al (2010) Caveolin-1 knockout mice exhibit impaired induction of mGluR-dependent long-term depression at CA3-CA1 synapses. Proc Natl Acad Sci U S A 107: 21778–21783.2109866210.1073/pnas.1015553107PMC3003045

[4] BehlC (2002) Estrogen can protect neurons: modes of action. J Steroid Biochem Mol Biol 83: 195–197.1265071610.1016/s0960-0760(02)00271-6

[5] OkadaM, MuraseK, MakinoA, NakajimaM, KakuT, et al (2008) Effects of estrogens on proliferation and differentiation of neural stem/progenitor cells. Biomed Res. 29: 163–170.10.2220/biomedres.29.16318614850

[6] Jung-TestasI, RenoirM, BugnardH, GreeneGL, BaulieuEE (1992) Demonstration of steroid hormone receptors and steroid action in primary cultures of rat glial cells. J Steroid Biochem Mol Biol 41: 621–631.156253310.1016/0960-0760(92)90394-x

[7] FesterL, Ribeiro-GouveiaV, Prange-KielJ, von SchassenC, BöttnerM, et al (2006) Proliferation and apoptosis of hippocampal granule cells require local oestrogen synthesis. J Neurochem 97: 1136–1144.1657983310.1111/j.1471-4159.2006.03809.x

[8] ArevaloMA, Santos-GalindoM, BelliniMJ, AzcoitiaI, Garcia-SeguraLM (2010) Actions of estrogens on glial cells: Implications for neuroprotection. Biochim Biophys Acta 1800: 1106–1112.1981838410.1016/j.bbagen.2009.10.002

[9] BarhaCK, GaleaLA (2010) Influence of different estrogens on neuroplasticity and cognition in the hippocampus. Biochim Biophys Acta 1800: 1056–1067.2010054510.1016/j.bbagen.2010.01.006

[10] FiocchettiM, AscenziP, MarinoM (2012) Neuroprotective effects of 17β-estradiol rely on estrogen receptor membrane initiated signals. Front Physiol 3: 73.2249358310.3389/fphys.2012.00073PMC3319910

[11] Zhang QG, Wang R, Tang H, Dong Y, Chan A, et al.. (2014) Brain-Derived Estrogen Exerts Anti-inflammatory and Neuroprotective Actions in the Rat Hippocampus. Mol Cell Endocrinol pii: S0303-7207(14)00036-7.10.1016/j.mce.2013.12.019PMC404031324508637

[12] BourqueM, DluzenDE, Di PaoloT (2009) Neuroprotective actions of sex steroids in Parkinson’s disease. Front Neuroendocrinol 30: 142–157.1941059710.1016/j.yfrne.2009.04.014

[13] LuchettiS, HuitingaI, SwaabDF (2011) Neurosteroid and GABA-A receptor alterations in Alzheimer’s disease, Parkinson’s disease and multiple sclerosis. Neuroscience 191: 6–21.2151436610.1016/j.neuroscience.2011.04.010

[14] LebesgueD, ChevaleyreV, ZukinRS, EtgenAM (2009) Estradiol rescues neurons from global ischemia-induced cell death: multiple cellular pathways of neuroprotection. Steroids 74: 555–561.1942844410.1016/j.steroids.2009.01.003PMC3029071

[15] MaggiA (2011) Liganded and unliganded activation of estrogen receptor and hormone replacement therapies. Biochim Biophys Acta 1812: 1054–1060.2160566610.1016/j.bbadis.2011.05.001PMC3121051

[16] CastoriaG, MigliaccioA, GiovannelliP, AuricchioF (2010) Cell proliferation regulated by estradiol receptor: Therapeutic implications. Steroids 75: 524–527.1987988910.1016/j.steroids.2009.10.007

[17] NilssonS, GustafssonJÅ (2011) Estrogen receptors: therapies targeted to receptor subtypes. Clin Pharmacol Ther 89: 44–55.2112431110.1038/clpt.2010.226

[18] SchlegelA, WangC, PestellRG, LisantiMP (2001) Ligand-independent activation of oestrogen receptor alpha by caveolin-1. Biochem J 359: 203–210.1156398410.1042/0264-6021:3590203PMC1222136

[19] SimonsK, GerlMJ (2010) Revitalizing membrane rafts: new tools and insights. Nat Rev Mol Cell Biol 11: 688–699.2086187910.1038/nrm2977

[20] GaudreaultSB, BlainJF, GrattonJP, PoirierJ (2005) A role for caveolin-1 in post-injury reactive neuronal plasticity. J Neurochem 92: 831–839.1568648510.1111/j.1471-4159.2004.02917.x

[21] SrivastavaDP, WatersEM, MermelsteinPG, KramárEA, ShorsTJ, et al (2011) Rapid estrogen signaling in the brain: implications for the fine-tuning of neuronal circuitry. J Neurosci 31: 16056–16063.2207265610.1523/JNEUROSCI.4097-11.2011PMC3245715

[22] HeadBP, PeartJN, PanneerselvamM, YokoyamaT, PearnML, et al (2010) Loss of caveolin-1 accelerates neurodegeneration and aging. PLoS One 5: e15697.2120346910.1371/journal.pone.0015697PMC3009734

[23] BiR, BroutmanG, FoyMR, ThompsonRF, BaudryM (2000) The tyrosine kinase and mitogen-activated protein kinase pathways mediate multiple effects of estrogen in hippocampus. Proc Natl Acad Sci U S A 97: 3602–3607.1072538310.1073/pnas.060034497PMC16286

[24] Colucci-D’AmatoGL, TinoA, Pernas-AlonsoR, ffrench-MullenJMH, di PorzioU (1999) Neuronal and glial properties coexist in a novel mouse CNS immortalized cell line. Exp Cell Res 252: 383–391.1052762810.1006/excr.1999.4636

[25] ChamberyA, Colucci-D’AmatoL, VissersJP, ScarpellaS, LangridgeJI, et al (2009) Proteomic profiling of proliferating and differentiated neural mes-c-myc A1 cell line from mouse embryonic mesencephalon by LC-MS. J Proteome Res 8: 227–238.1907224110.1021/pr800454n

[26] SeverinoV, FarinaA, Colucci-D’AmatoL, RecciaMG, VolpicelliF, et al (2013) Secretome profiling of differentiated neural mes-c-myc A1 cell line endowed with stem cell properties. Biochim Biophys Acta 1834: 2385–2395.2324671210.1016/j.bbapap.2012.12.005

[27] VolpicelliF, ConsalesC, CaiazzoM, Colucci-D’AmatoL, Perrone-CapanoC, et al (2004) Enhancement of dopaminergic differentiation in proliferating midbrain neuroblasts by sonic hedgehog and ascorbic acid. Neural Plast 11: 45–57.1530330510.1155/NP.2004.45PMC2565440

[28] VolpicelliF, Perrone-CapanoC, Da PozzoP, Colucci-D’AmatoL, di PorzioU (2004) Modulation of nurr1 gene expression in mesencephalic dopaminergic neurones. J Neurochem 88: 1283–1294.1500968410.1046/j.1471-4159.2003.02254.x

[29] SchmittgenTD, LivakKJ (2008) Analyzing real-time PCR data by the comparative. Nat Protoc 3: 1101–1108.1854660110.1038/nprot.2008.73

[30] GrecoD, VolpicelliF, Di LietoA, LeoD, Perrone-CapanoC, et al (2009) Comparison of gene expression profile in embryonic mesencephalon and neuronal primary cultures. PLoS One 4: e4977.1930550310.1371/journal.pone.0004977PMC2654915

[31] MigliaccioA, CastoriaG, Di DomenicoM, de FalcoA, BilancioA, et al (2002) Sex steroid hormones act as growth factors. J Steroid Biochem Mol Biol 83: 31–35.1265069910.1016/s0960-0760(02)00264-9

[32] PeiroS, ComellaJX, EnrichC, Martin-ZancaD, RocamoraN (2000) PC12 cells have caveolae that contain TrkA. Caveolae-disrupting drugs inhibit nerve growth factor-induced, but not epidermal growth factor-induced, MAPK phosphorylation. J Biol Chem 275: 37846–37852.1098278810.1074/jbc.M000487200

[33] RaabH, KarolczakM, ReisertI, BeyerC (1999) Ontogenetic expression and splicing of estrogen receptor-alpha and beta mRNA in the rat midbrain. Neurosci Lett 275: 21–24.1055497510.1016/s0304-3940(99)00723-5

[34] KüppersE, BeyerC (1999) Expression of estrogen receptor-alpha and beta mRNA in the developing and adult mouse striatum. Neurosci Lett 276: 95–98.1062480010.1016/s0304-3940(99)00815-0

[35] CordeyM, PikeCJ (2005) Neuroprotective properties of selective estrogen receptor agonists in cultured neurons. Brain Res 1045: 217–223.1591078010.1016/j.brainres.2005.03.032

[36] DubalDB, ZhuH, YuJ, RauSW, ShughruePJ, et al (2001) Estrogen receptor alpha, not beta, is a critical link in estradiol-mediated protection against brain injury. Proc Natl Acad Sci U S A 98: 1952–1957.1117205710.1073/pnas.041483198PMC29363

[37] PatroneC, PollioG, VegetoE, EnmarkE, de CurtisI, et al (2000) Estradiol induces differential neuronal phenotypes by activating estrogen receptor alpha or beta. Endocrinology 141: 1839–1845.1080359410.1210/endo.141.5.7443

[38] DubalDB, RauSW, ShughruePJ, ZhuH, YuJ, et al (2006) Differential modulation of estrogen receptors (ERs) in ischemic brain injury: a role for ERalpha in estradiol-mediated protection against delayed cell death. Endocrinology 147: 3076–3084.1652784810.1210/en.2005-1177

[39] AcconciaF, TottaP, OgawaS, CardilloI, InoueS, et al (2005) Survival versus apoptotic 17beta-estradiol effect: role of ER alpha and ER beta activated non-genomic signaling. J Cell Physiol 203: 193–201.1538962710.1002/jcp.20219

[40] Zhang QG, Wang R, Tang H, Dong Y, Chan A, et al.. (2014) Brain-Derived Estrogen Exerts Anti-inflammatory and Neuroprotective Actions in the Rat Hippocampus. Mol Cell Endocrinol pii: S0303-7207(14)00036-7.10.1016/j.mce.2013.12.019PMC404031324508637

[41] GalbiatiF, RafaniB, LisantiMP (2001) Emergine themes in lipid rafts and caveolae. Cell 106: 403–411.1152572710.1016/s0092-8674(01)00472-x

[42] ShenJ, MaS, ChanP, LeeW, FungPC, et al (2006) Nitric oxide down-regulates caveolin-1 expression in rat brains during focal cerebral ischemia and reperfusion injury. J Neurochem 96: 1078–1089.1641758710.1111/j.1471-4159.2005.03589.x

[43] GaudreaultSB, DeaD, PoirierJ (2004) Increased caveolin-1 expression in Alzheimer’s disease brain. Neurobiol Aging 25: 753–759.1516570010.1016/j.neurobiolaging.2003.07.004

[44] BoschM, MaríM, HermsA, FernándezA, FajardoA, et al (2011) Caveolin-1 deficiency causes cholesterol-dependent mitochondrial dysfunction and apoptotic susceptibility. Curr Biol 21: 681–686.2149709010.1016/j.cub.2011.03.030PMC3409647

[45] FraAM, WilliamsonE, SimonsK, PartonRG (1995) De novo formation of caveolae in lymphocytes by expression of VIP21-caveolin. Proc Natl Acad Sci USA 92: 8655–8659.756799210.1073/pnas.92.19.8655PMC41025

[46] OkamotoT, LisantiMP, EngelmanJA, WykoffCC, YasuharaS, et al (1997) Recombinant expression of caveolin-1 in oncogenically transformed cells abrogates anchorage-independent growth. J Biol Chem 272: 16374–16381.919594410.1074/jbc.272.26.16374

[47] HeadBP, PatelHH, TsutsumiYM, HuY, MejiaT, et al (2008) Caveolin-1 expression is essential for N-methyl-D-aspartate receptor-mediated Src and extracellular signal-regulated kinase 1/2 activation and protection of primary neurons from ischemic cell death. FASEB J 22: 828–840.1790572410.1096/fj.07-9299com

[48] HeadBP, HuY, FinleyJC, SaldanaMD, BondsJA, et al (2011) Neuron-targeted caveolin-1 protein enhances signaling and promotes arborization of primary neurons. J Biol Chem 286: 33310–33321.2179901010.1074/jbc.M111.255976PMC3190943

[49] BrunaldiK, HuangN, HamiltonJA (2010) Fatty acids are rapidly delivered to and extracted from membranes by methyl-beta-cyclodextrin. J Lipid Res 51: 120–131.1962573510.1194/jlr.M900200-JLR200PMC2789772

[50] CowleyS, PatersonH, KempP, MarshallCJ (1994) Activation of MAP kinase kinase is necessary and sufficient for PC12 differentiation and for transformation of NIH 3T3 cells. Cell 77: 841–852.791173910.1016/0092-8674(94)90133-3

[51] Colucci-D’AmatoL, Perrone-CapanoC, di PorzioU (2003) Chronic activation of ERK and neurodegenerative diseases. Bioessays 25: 1085–1095.1457924910.1002/bies.10355

[52] StanciuM, WangY, KentorR, BurkeN, WatkinsS, et al (2000) Persistent activation of ERK contributes to glutamate-induced oxidative toxicity in a neuronal cell line and primary cortical neuron cultures. J Biol Chem 275: 12200–12206.1076685610.1074/jbc.275.16.12200

[53] Colucci-D’AmatoGL, D’AlessioA, CalifanoD, CalìG, RizzoC, et al (2000) Abrogation of Nerve Growth Factor-induced terminal differentiation by ret oncogene involves perturbation of nuclear translocation of ERK. J Biol Chem 275: 19306–19314.1085845910.1074/jbc.275.25.19306

[54] IndrigoM, PapaleA, OrellanaD, BrambillaR (2010) Lentiviral vectors to study the differential function of ERK1 and ERK2 MAP kinases. Methods Mol Biol 661: 205–220.2081198510.1007/978-1-60761-795-2_12

[55] GarnierM, Di LorenzoD, AlbertiniA, MaggiA (1997) Identification of estrogen-responsive genes in neuroblastoma SK-ER3 cells. J Neurosci 17: 4591–4599.916952010.1523/JNEUROSCI.17-12-04591.1997PMC6573342

[56] LiuJ, WangXB, ParkDS, LisantiMP (2002) Caveolin-1 expression enhances endothelial capillary tubule formation. J Biol Chem 277: 10661–10668.1174823610.1074/jbc.M110354200

[57] PodarK, TaiYT, ColeCE, HideshimaT, SattlerM, et al (2003) Essential role of caveolae in interleukin-6 and insulin-like growth factor I-triggered Akt-1-mediated survival of multiple myeloma cells. J Biol Chem 278: 5794–5801.1248287810.1074/jbc.M208636200

